The article "Neuronal and glial changes in the brain resulting from explosive blast in an experimental model" was published in 2016. Journal: Acta Neuropathol Commun.

# Neuronal and glial changes in the brain resulting from explosive blast in an experimental model

**DOI:** 10.1186/s40478-016-0395-3

**Published:** 2016-11-24

**Authors:** James A. Goodrich, Jung H. Kim, Robert Situ, Wesley Taylor, Ted Westmoreland, Fu Du, Steven Parks, Geoffrey Ling, Jung Y. Hwang, Amedeo Rapuano, Faris A. Bandak, Nihal C. de Lanerolle

**Affiliations:** 1 Department of Comparative Medicine, Yale School of Medicine, New Haven, CT USA; 2 Department of Pathology, Yale School of Medicine, New Haven, CT USA; 3 Department of Neurosurgery, Yale School of Medicine, 333 Cedar Street, New Haven, CT 06520-8082 USA; 4 Advanced Medical Training, McKinney, TX USA; 5 FD NeuroTechnologies Inc., Ellicott City, MD USA; 6 ORA Inc, Fredericksburg, VA USA; 7 Department of Neurology, Edward Hébert School of Medicine, Uniformed Services University of the Health Sciences, Bethesda, MD USA; 8 Integrated Services Group Inc., Potomac, MD USA

## Abstract

Mild traumatic brain injury (mTBI) is the signature injury in warfighters exposed to explosive blasts. The pathology underlying mTBI is poorly understood, as this condition is rarely fatal and thus postmortem brains are difficult to obtain for neuropathological studies. Here we report on studies of an experimental model with a gyrencephalic brain that is exposed to single and multiple explosive blast pressure waves. To determine injuries to the brain resulting from the primary blast, experimental conditions were controlled to eliminate any secondary or tertiary injury from blasts. We found small but significant levels of neuronal loss in the hippocampus, a brain area that is important for cognitive functions. Furthermore, neuronal loss increased with multiple blasts and the degree of neuronal injury worsened with time post-blast. This is consistent with our findings in the blast-exposed human brain based on magnetic resonance spectroscopic imaging. The studies on this experimental model thus confirm what has been presumed to be the case with the warfighter, namely that exposure to multiple blasts causes increased brain injury. Additionally, as in other studies of both explosive blast as well as closed head mTBI, we found astrocyte activation. Activated microglia were also prominent in white matter tracts, particularly in animals exposed to multiple blasts and at long post-blast intervals, even though injured axons (i.e. β-APP positive) were not found in these areas. Microglial activation appears to be a delayed response, though whether they may contribute to inflammation related injury mechanism at even longer post-blast times than we tested here, remains to be explored. Petechial hemorrhages or other gross signs of vascular injury were not observed in our study. These findings confirm the development of neuropathological changes due to blast exposure. The activation of astrocytes and microglia, cell types potentially involved in inflammatory processes, suggest an important area for future study.

## Introduction

Exposure to explosive blast pressure waves is thought to cause mild traumatic brain injury (mTBI) in warfighters [20]. However, little is known of the neuropathological changes in the brain resulting from exposure to blast. Injury to axons caused in traumatic brain injury (TBI) has received considerable attention [2, 12], though studies of neuronal and non-neuronal cells in mTBI are more limited. This is particularly so in explosive blast trauma as mTBI is rarely fatal and thus post-mortem brains are not readily available for histopathological investigation.

Imaging studies on patients with mTBI from blast have been conducted to assess injury to the brain. While standard magnetic resonance imaging studies have failed to observe any evidence of cellular injury [12], magnetic resonance spectroscopic imaging (MRSI) studies have proven more useful. MRSI studies focus on the measurement of millimolar concentrations of low molecular weight molecules. These molecules include N-acetyl-acetate (NAA), a compound found only in neurons [32], and reductions in NAA are typically interpreted to reflect neuronal loss or injury. In contrast, choline (Ch) is a trimethylamine, that is associated with axon membrane damage and repair [4], and increases in choline are seen in diseases that result in axonal damage [12]. Creatine (Cr), both phosphorylated and un-phosphorylated forms of phosphocreatine that is the primary buffer for ATP requiring processes [12] is also used as a measure of mitochondrial metabolic injury. MRSI studies, done on veterans exposed to explosive blast and with a history of self-reported memory impairment, found significant reductions in the ratio of NAA/Ch and NAA/Cr in the anterior hippocampus. Metabolite ratio reductions in the right hippocampus were more extensive than in the left. Hippocampal volume measurements revealed that the right hippocampus was about 20% smaller than the left [6]. These findings suggest neuronal injury in the hippocampus. The changes were independent of co-morbidities such as PTSD and depression [6, 11, 12] but associated with reductions in visual memory [6]. These findings suggest neuronal injury in the hippocampus. In order to establish if such changes in metabolite ratios are associated with neuronal and other cellular changes in the brain, the histopathology of the brain of Yorkshire swine exposed to explosive blast pressure waves in operationally relevant situations was studied at two weeks post blast [5]. This study did not show evidence of neuronal injury but did reveal significant astrocyte and microglial activation [5].

In this paper we report the neuronal and glial changes in the brains of Yucatan minipigs exposed to pure explosive blast waves that survived for longer periods, 6 to 8 months post blast. We also report on the effects of single, double and triple blast exposure. We found significant neuronal injury in the hippocampus with longer post-blast intervals. In addition, there was also significant astrocyte and microglial activation and proliferation.

## Material and methods

### Subjects

The animals utilized in this study were intact male naïve Yucatan Minipigs (*Sus scrofa domestica*) (Age mean 6.9 SD ± 4 months, Median 5 months; *n* = 45) supplied by Sinclair Bio-resources of Columbia, Missouri from their Windham, Maine and Missouri herds. The herd is maintained at a biosecurity level to exclude most common swine pathogens as indicated on their website http://www.sinclairbioresources.com. The Yale, ACI-AMT, and DOD (ACURO) Institutional Animal Care and Use Committees (IACUCs) approved all aspects of the described studies. Both animal care programs have full AAALAC accreditation.

Upon purchase, the animals were entered into an acclimation protocol consisting of a minimum of 4-days residency at the animal care facility prior to experimentation. During this time they were treated prophylactically with fenbendazole (PO) and ceftiofur sodium (IM). The pigs were housed in barrier isolation from pigs derived from other sources and fed Teklad Miniswine diet 7037 and had access to water through automatic valves ad libitum. Group housing was used when feasible but individual housing was required to prevent fighting as the all-male group matured. Environmental enrichment included daily access to toys, fruit and vegetables and regular exercise outside the pen enabling social interaction with the other pigs and care staff. The light cycle was 12 h of light and 12 h of darkness. And the room temperatures were maintained at 72° ±2 °F and approximately 15 air changes per hour. Pens were bedded with wood chips and the square footage of floor space met or exceeded guidelines in the ILAR Guide for the Care and Use of Laboratory Animals based on body weight.

### Animal preparation for experimental blast exposure

Each animal (except controls) was anesthetized for the blast exposure procedure. Initially, each pig was injected intramuscularly with a combination of Telazol (4.4 mg/kg) and ketamine (5-10 mg/kg) and buprenorphine (0.3 mg/pig). After the telazol/ketamine induction, an intravenous catheter (18–22 ga, 1–1.5″) was placed in an ear vein and endotracheal intubation was achieved with a 6.0–8.0 cuffed endotracheal tube. Dexmedetomidine at 5–20 μg/kg was given IM or IV to assist in intubation and analgesia. Glycopyrrolate (0.01 mg/kg IM/IV) was given at this time to minimize cardiovascular depression during anesthesia. Ventilation was provided manually as needed with ambient air via an ambu-bag manual ventilator.

Midazolam (0.2–0.3 mg/kg q15–30 min) was utilized to minimize anxiety and assist in sedation from the transportation phase through recovery. Anesthesia was maintained with IV or IM boluses of Ketamine (3–5 mg/kg q15–30 min), and one or a combination of the following: Dexmedetomidine (4–10 μg/kg q60–90 min), Midazolam (0.2–0.3 mg/kg q15–30 min). During anesthesia and the blast procedures, monitoring consisted of chest and cardiac auscultation, assessment of jaw tone, palpebral and corneal reflexes, withdrawal from toe or ear pinch, reaction to surgical stimulation, and the utilization of pulse oximetry and EKG electronic monitoring devices. A Bluetooth-enabled physiology monitor was connected to each animal throughout induction, preparation, blast and recovery.

### Explosive blast exposure

Upon reaching a surgical plane of anesthesia, each pig was placed in sternal recumbency, then wrapped in specially made Kevlar and lead body protection with a stockinette over the head to keep the eyes shut and protect the face. Once the blast protective wrap was in place, the entire animal was wrapped in a leather overwrap and a heavy gauge web sling that covered the entire animal from rump to snout. The animal was then positioned in the experimental chamber and attached to a support frame.

Exposure to blast was carried out in a 3-wall test structure [5]. The animal was positioned with its head in the right rear corner, oriented 45° facing the walls. The explosive charge was suspended overhead. Liquid NitromethaneTriethanolamine (98%) was used to generate the explosion. The charge was to the rear left of the animal and was chosen after preliminary dose calibration trials to determine the maximum dose that did not cause physical injury to the body. An average pressure of 100 psi was generated near the head. Separate groups of animals were exposed to single (*n* = 16), double (*n* = 15) and triple (*n* = 3) blast exposures; the second and third exposures occurred a week apart. Within minutes after exposure to explosion, the animal was removed from the support frame and taken to a nearby facility for recovery. All physiological parameters were monitored until full recovery and endotracheal tube removal. Pulmonary injury immediately after blast was assessed clinically by the following signs: 1) blood from the respiratory tract post-blast exposure, 2) changes in lung sounds post-blast, 3) respiratory distress during recovery, and 4) coughing post-blast with no concurrent evidence of infectious disease in the individual or cohort group. The severity of blast lung from the explosive levels used for this study was quantified as follows: 0, no blast lung signs (i.e no blood from respiratory tract, lungs clear); 1, mild (small amount of blood, 0–3 ml and mild increased respiratory sounds); 2, moderate (moderate or significant blood, 3–10 ml, increased lung sounds with respiratory distress at recovery and coughing post-blast; 3, severe (significant blood, severe lung sounds, severe distress or died during recovery). In our study overall only 12% of the animals exhibited a level 2 or 3 pulmonary injury and were not included in these neuropathological studies. Exposure to a second or third blast did not increase clinical blast lung scores. Only the animals exposed to a single, double and triple-blasts and had clinical scores of 0 or 1, were chosen for our study.

Buprenorphine, administered intravenously, was repeated every 6 h for 12–48 h post-blast to provide opioid analgesic value. Animals were given a general neurological examination immediately after recovery and about 2 weeks later. No neurological deficits were detected during the post-blast survival period.

The definition of “mild” traumatic brain injury in human studies is based on clinical signs involving the period of post blast loss of consciousness and post blast amnesia. Since our animals were under sedation and anesthetized when exposed to blast (required for animal welfare reasons), post blast loss of consciousness could not be determined, and since the animals took a few hours to recover from anesthesia, post blast amnesia was not determined. Thus our working definition of “mild” TBI in this study was based on the fact that the blast exposure did not result in any overt signs such as injury to skull or intracranial hemorrhage (established during neuropathology), and their assumption of normal behavior (feeding, locomotion etc.) once recovered from anesthesia. Additionally as detailed below, neuronal density assessments show significant but mild neuronal loss.

### Histology

Following periods of post-blast survival ranging from 2 weeks to 8 months, the animals were sacrificed to harvest their brains for histological investigation. To this end, anesthesia was induced in each pig with a combination of tiletamine-zolazepam, ketamine, xylazine and atropine and masked with isoflurane for placement of an ear vein catheter and endotracheal intubation and maintained on isoflurane. Buprenorphine and 20,000 units of Heparin were administered intravenously, a fentanyl continuous rate intravenous infusion was added and the isoflurane was increased 4–5% from maintenance levels followed by intravenous lidocaine to produce multi-modal analgesia. Next the brain was rapidly perfused in situ, via cardiac left ventricular access, with 1 l of cold phosphate buffered saline, followed by 1 l of 1% paraformaldehyde and then 3-6 l of Zamboni’s fixative [31], all under mechanical pump pressure. The animals head was left undisturbed for 20–24 h at 4 °C (to continue in situ fixation and eliminate handling artifacts) before the brain was removed from the skull and stored in Zamboni’s solution. Each brain was then weighed, sliced into 2 mm cross-sections, photographed and stored in Zamboni’s solution for two weeks until it was processed for histological sectioning.

The pathology was evaluated at four levels through the neuraxis of the brain – 1) prefrontal cortex; 2) frontal cortex, basal ganglia and thalamus including the internal capsule, corpus callosum as well as portions of the lateral and third ventricle; 3) hippocampus, the amygdala and the thalamus or midbrain; 4) cerebellum and medulla. Six-micrometer thick paraffin embedded sections were cut in the coronal plane. Twenty serial sections were mounted on individual microscope slides and stored at room temperature before further processing. Adjacent sections from each block were subjected to the following staining procedures. Hematoxylin and eosin (H& E) staining (FD Neurotechnologies Inc.), and Flurojade B staining (Histochem, Jefferson, AR) was carried out according to standard staining procedures. Deparaffinized sections were immunostained using the following specific primary antibodies: rabbit anti-glial fibrillary acidic protein (GFAP, 1:600; Dako, Carpinteria, CA), rabbit anti-C-terminus of the human β-amyloid precursor protein (β-APP, 1:200; Invitrogen, Carlsbad, CA), rabbit anti-ionized calcium-binding adaptor molecule 1 (Iba1, 1:1000 Wako Chemicals USA, Richmond, VA), mouse anti-phospho-PHF-tau pSer202 + Thr205 (AT8, 1:100, Thermo Fisher Scientific, Rockford, IL.), rabbit anti-amyloid beta (1–42) (1:100, Life Technologies, Grand Island, NY). The bound antibodies were visualized using the avidin-biotin complex method with the Vectastain elite ABC kit (Vector, Burlingame, CA). In brief, sections were incubated in PBS containing Triton X-100, blocking serum, and a biotinylated secondary antibody for 1 h and then in PBS containing an avidin-biotinylated horseradish peroxidase complex for1 h. This was followed by incubation of the sections for 10 min in 0.05 mol/L Tris buffer (pH 7.2) containing 0.03% 3’,3’-diaminobenzidine (Sigma) and 0.0075% H_2_O_2_. After thorough rinses in distilled water, sections were dehydrated in ethanol, cleared in xylene, and coverslipped in Permount.

### Quantitation of cellular changes

The methods used are the same as those in a previous study [5, 18]. Neuronal counts were determined in 6 μm thick paraffin sections stained with Hematoxylin and eosin. A trained technician performed the neuronal counts blind to the treatment condition of the animal. The hippocampus was divided into CA1 through CA4 and dentate granular layer according to Lorente de No [23] (Fig. 1), and a modified method of Mouritzen Dam was utilized for neuronal counting [25]. Neuronal nuclei were counted in each unit area of a 100-μm × 200-μm rectangle for CAI through CA4 fields and a 50-μm × 100-μm rectangle for the dentate granular layer, using an ocular grid calibrated with a stage micrometer. CA fields and the dentate granular layer were covered with multiple continuous unit areas through the ocular grid as counting was performed. The neuronal numbers obtained were adjusted with the Abercrombie’s formula [1] utilizing 8 μm for the nuclear diameter of pyramidal neurons and 6 μm for that of granular neurons, and neuronal density was expressed as mean neuronal number/mm^3^. The Kruskal-Wallis one-way analysis of variance test [29] was utilized to determine that neuronal densities among the control, single blast, double blast and triple blast were from different populations. To compare the statistical differences in neuronal density for pairwise comparisons the Mann-Whitney U, 2-tailed test was used [29]. The data of the latter were interpreted after the application of Bonferroni’s procedure for multiple testing.

**Fig. 1:** Coronal sections through the hippocampus of a Yucatan Minipigs, *Top* Control. *Bottom* Blast exposed. They are stained with Haematoxylin and Eosin to illustrate hippocampal subregions in which neurons were quantified. CA1, CA2 and CA3 are subregions of the *Cornu Ammonis* (Ammon’s horn) with arrows that indicate their boundaries. GC, dentate granule cell layer. H, dentate hilus. ML, dentate molecular layer. Scale bar = 500 μm

Astrocytes were counted in anti-GFAP stained 6 μm thick sections using a modification of the optical fractionator method of Stereo Investigator (MicroBrightfield, Inc., Williston, VT). In brief, the regions in which astrocytes were counted were traced out by drawing closed contours around them. A counting frame of 200 μm × 200 μm was chosen, and the first area to be counted within the defined region was randomly selected by a software program, based off the upper left corner of the defined region. Twenty randomly selected sites were chosen for counting. All astrocyte cell bodies with visible nuclei within each counting frame were enumerated, and the number of astrocytes per square millimeter was calculated from the 20 areas sampled within the defined region. Counts were done in the dentate molecular layer and hilus on two sections at each level showing the hippocampus and data were averaged per animal. Statistically significant differences between treatment groups were determined with the Mann-Whitney 2-tailed test.

## Results

### Patterns of neuronal density in the hippocampus

We first sought to determine the best dose of explosive required for mild brain injury without incapacitating the animals so they could survive longer to study the development of injury with time. Thus, 15 swine were exposed to single blasts at three levels of explosive blast pressures (*n* = 7 at 70 psi, *n* = 4 at 100 psi and *n* = 5 at 130 psi). The animals in this calibration study survived post-blast for about a month (mean 25 ± 6 days). Neuronal counts were determined in the sub-fields of the hippocampus (dentate gyrus, hilus, CA3/2 and CA1) separately for the left (blast exposed side) and right side. Comparison of neuronal densities in CA1 between the three groups in the calibration study did not show any significant difference and thus they were combined for comparison with other test groups. Comparison of neuronal counts on the two sides of the brain for the controls and for each blast exposure group showed no significant differences, and thus the average for the two sides in each sub-field was used for further intergroup comparisons. Pairwise comparisons between groups were made (Mann-Whitney *U* test) as there were overall significant differences between groups (Kruskal-Wallis one-way analysis of variance test), (Table 1).

**Table 1:** Neuron densities number per mm^3^

Group		CA1	CA2-3	CA4	Dentate
Control	Mean	192.08	180.14	78.74	1535.7
*n* = 11	± SD	27.32	39.26	12.47	134.05
Single blast	Mean	181.08	174.97	76.44	1461.82
*n* = 16	± SD	26.53	36.46	14.47	98.03
Double blast	Mean	167.43	176.91	69.97	1467.26
*n* = 15	± SD	24.25	43.71	9.3	158.38
Triple blast	Mean	149.15	153.59	67.32	1560.9
*n* = 3	± SD	10.08	34.07	12.3	124.31
All blast	Mean	171.98	174.72	72.61	1473.48
	± SD	26.08	39.62	12.45	132.57
Control vs single	*p*	ns	ns	ns	0.0092
Control vs Double	*p*	0.0005	ns	0.0126	0.0266
Control vs Triple	*p*	0.0013	ns	0.0802	ns
Control vs All	*p*	0.0004	ns	0.0385	ns
single vs Double	*p*	0.018	ns	0.07	ns
Single vs Triple	*p*	0.002	ns	0.13	ns
Double vs Triple	*p*	0.032	ns	ns	ns

The intergroup significance values are derived from the Mann-Whitney *U*-test, two tail. CA = neurons in the pyramidal layer of Cornu Ammonis (Ammon’s Horn) areas 1 to 4 of the hippocampus. Dentate = neuron densities in the dentate granule cell layer

A comparison of neuronal densities of hippocampal sub-fields of controls and single blast exposed animals indicated a significant loss of neurons only in the dentate gyrus. A similar comparison between controls and animals subjected to two blast-exposures (double exposure group) revealed significant neuronal loss in CA1 and the hilus (CA4) in addition to the dentate gyrus (Table 1) Neuronal loss was also observed in CA1 and the hilus but not the dentate gyrus in the triple blast-exposed group compared to controls. A comparison of all blast-exposed animals as one group with the controls also revealed significant neuronal loss the CA1 and the hilus (CA4). Compared to single blast exposed animals, double and triple blast-exposed animals showed greater neuronal loss in CA1, but not significantly in the hilus. Thus, CA1 appears to be most sensitive to blast pressure wave injury.

As the animals in the single exposure group were exposed to blast pressures generated from three different doses of explosives, we examined the overall differences in neuron densities with particular blast pressures or no blast (controls) (Kruskal-Wallis analysis of variance [29]), This analysis showed no differences at about the one month post-blast time point (*n* = 21, *H* = 1.610, not significant). Since animals were inducted into the studies at a median age of 5 months and were maintained post-blast for varying periods of time, during which they continued to grow, we queried the possible correlations of age, weight and post-blast survival period at the point of sacrifice, with neuronal densities in CA1, (Table 1), regardless of blast exposure paradigms. The application of the Spearman Rank Correlation Coefficient test showed significant negative correlations between neuronal densities and animal weight (r_s_ −0.409832, *p* ≤ 0.05), age (r_s_ −0.3585721, *p* ≤ 0.05) and post-blast survival period (r_s_ −0.54780, 0.01 > *p* > 0.005).

### Patterns of astrocyte activation

Astrocyte activation and proliferation was assessed by immunostaining for GFAP and was a prominent feature in the blast-exposed swine brain. This was readily seen by visual observation of the dentate hilus and molecular layer of the hippocampus (Fig. 2a) and in CA1 (Fig. 2b). Astrocyte densities were determined for the dentate hilus and molecular layer areas of the hippocampus to assess the relationship between astrocyte activation and blast exposure. The densities were first determined for left and right hippocampi separately. As there were no statistical differences between the two sides, the average of values for both sides were used to compare groups of animals with varying blast exposure patterns (Table 2). An analysis of variance performed on density measurements of all animals in all exposure groups showed that there were differences between groups (*p* < 0.001, Kruskal-Wallis one-way analysis of variance test). Pairwise group comparisons revealed that animals subjected to single blast exposure had significantly higher densities of astrocytes in both the hilus and molecular layer than sham controls (Table 2). Similarly, animals exposed to two blasts had significantly higher densities of astrocytes compared to those exposed to a single blast in both regions. The astrocyte densities in double blast-exposed animals were almost doubled that of the control animals (Table 2). Whereas animals exposed to triple blasts had significantly higher densities than those exposed to a single blast, there were no differences between double and triple blast. This latter observation may in part be due to the small number of animals (*n* = 3) in the triple blast group. The activated and new astrocytes in the single and double blast-exposed animals were strongly immunoreactive for GFAP and had a distinctive stellate appearance, with the processes of adjacent astrocytes not overlapping and maintaining a tiled appearance [5]. This morphology is in contrast to that of astrocytes that are described for areas of high neuronal injury where their processes interdigitate. The triple blast-exposed animals showed astrocyte proliferation and activation in the deep central white matter in addition to the hippocampus (Fig. 3b). The astrocytes often appeared swollen and intensely reactive for GFAP (gemistocytic astrocytes) (Fig. 3b). Astrocyte activation and proliferation in the hippocampus was detected at the earliest time point evaluated, 2 weeks, and remained still present even at 6–8 months post blast.

**Fig. 2:** Photomicrographs of hippocampal sections immunostained for GFAP an astrocyte marker. **a** An image through the polymorphic layer, granule cell layer and the molecular layer of the dentate gyrus, showing increased immunoreactivity the blast exposed animal compared to a control. **b** A portion of area CA1 showing increased immunoreactivity and proliferation of astrocytes throughout the layers

**Table 2:** Astrocyte density, (number per mm^2^) ± SD in the dentate area

Treatment	Hilus per mm2	ML per mm2
Controls	7.588	5.857
*n* = 6	±0.863	±1.093
Single	10.118	8.469
*n* = 9	±0.538	±1.240
Double	12.691	11.035
*n* = 8	±1.282	±1.716
Triple	12.350	9.777
*n* = 3	±0.571	±0.554
Control vs. Single	*p* < 0 .002	*p* < 0.02
Single vs. Double	*p* < 0.002	*p* < 0.02
Single vs. Triple	*p* < 0.002	*p* < 0.05
Double vs. Triple	NS	NS

The intergroup significance values are derived with the Mann-Whitney U, two tail test. ML = dentate molecular layer. Treatment = number of blast exposures

**Fig. 3:** Photomicrographs of the deep central white matter area immunostained for GFAP showing astrocyte proliferation and activation, astrocytes often appearing swollen and intensely reactive for GFAP (gemistocytic astrocytes) in an animal exposed to triple blasts (**b**) compared to the same area in a non-blast exposed sham control (**a**)

### Patterns of microglial activation

The distribution of microglia was studied with Iba-1 immunostaining. Semi-quantitative assessments of Iba-1 stained cells were made in the gray matter areas (hippocampus, superior frontal cortex and thalamus) and white matter areas (corpus callosum and central white matter) in controls, single, double and triple blast exposed animals. Overall, activated microglia were not particularly noticeable in gray matter regions. There were noticeably few in the hippocampus and their patterns of distribution did not differ significantly between blast-exposed groups. Activated microglia, when observed, were mostly seen in the corpus callosum (Fig. 4) and central white matter. Morphological features of activated microglia, including swollen and elongated cell bodies with long extensions were detectable in the blast-exposed brains. The density of microglia appeared somewhat greater in triple blast exposed animals (Fig. 4). However, microglial activation was not present in every animal. Activated microglia were not seen at the 2-week and 1 month post-blast time points. The animals were usually 3 to 8 months post-blast when microglial activation was detected.

**Fig. 4:** Photomicrographs of the corpus callosum area in (**a**) a sham control, (**b**) animal exposed to a single blast, (**c**) animal exposed to double blast and (**d**) animal exposed to triple blasts and immunostained for Iba1 a marker for microglia. Activated microglia, which have elongated processes, swollen and somewhat elongated cell bodies and increased immunoreactivity are especially seen with (**c**) double and (**d**) triple blast animals

### Other markers

It has been reported that phosphorylated Tau expression is increased in humans subjected to traumatic brain injury [24] even explosive blast [9], resulting in a condition described as chronic traumatic encephalopathy (CTE). Hence, brain sections of swine exposed to varying levels of explosive blast and survived for up to 8 months post-blast, were stained immunohistochemically for either phosphorylated Tau (AT8 antibody) or beta Amyloid protein. Examination of the hippocampus, amygdala and frontal cortex showed no pathological expression of these molecules either in blast-exposed minipigs or controls. We specifically looked for, but found no tau-immunoreactive neurofibrillary tangles, astrocytic tangles, or accumulations of tau-immunoreactive astrocytes in perivascular locations even in swine that survived 6–8 months post-blast. Staining for beta-amyloid also did not show any differences between groups.

## Discussion

### Neuronal injury

In these studies on the Yucatan minipigs exposed to a single blast and examined about a month later, no significant neuron loss was detected. This result is similar to that of our previous study with domestic Yorkshire pigs exposed to a single explosive blast in three operationally relevant situations, where no evidence of neuronal loss was detected in hippocampus at a short (2 week) post-blast time point [5].

However, our data show a significant, though small level of neuronal loss resulting from exposure to double and triple blast. Loss is most significant in CA1 and the hilus of the hippocampus, suggesting that repeated blast-exposure results in greater neuronal injury. The present studies also examined the degree of neuronal injury at varying post-blast intervals after a single and multiple blasts, as opposed to only short post-blast intervals in our earlier study [5]. The longer post-blast survival periods correlate negatively with neuronal densities. Since such negative correlations were also observed with increased age and weight, the question arises as to whether these factors are responsible for the decrease in neuron densities. We think this is unlikely for several reasons. Minipigs have a life span of several years (12–15 years) with puberty around 3–5 month [10]. Thus, even at 8 months the pigs in our study are young adults. Further, it is shown that in Göttingen minipigs there is an increase, rather than decrease, in neuron density from 6–7 weeks to 8 months [10, 14]. A comparison of Göttingen minipigs and domestic pigs found no change in cortical neuronal densities from neonate (1–2 days) to adult (1.5–3 years) in domestic pigs. Thus, an increase in age over the range reported in this study would not result in neuronal loss. Additionally, a correlation analysis of age and gross brain weight for all the Yucatan minipigs included in this study irrespective of the blast exposure condition shows a significant positive linear correlation (R^2^ = 0.7358, y = 2.6736x + 76.035). This suggests an increase in cell numbers. Thus, there is a small but significant amount of neuronal loss in hippocampus (in CA1 ~ 10% loss with single blast, 13% with double blast and ~25% with triple blast). These data imply that small neuronal losses may be a feature of mild TBI. Such small losses in neuronal densities can only be detected by neuronal counts and are not visually observable.

Further, whereas the animals exposed to a single blast were allowed to survive for only about one month, those exposed to double and triple blasts were allowed to survive post-blast for 6 to 8 months. It may thus be argued that the additional neuronal loss in the latter two groups may be due the longer post-blast survival period rather than multiple blast exposures. While this remains a possibility, one of the double blast animals was survived for only 27 days and one of the triple blast animals for 40 days and their neuronal densities in CA1 were well within the range of the double and triple exposure groups. This provides evidence for the greater injury potential of multiple exposures. In MRSI studies done at both early (~1 month) and later time points (6–8 months) on the double and triple exposed animals (Hetherington et al., to be published), we were only able to detect evidence of neuronal injury in the hippocampus at the later time points. This provides further evidence of the importance of the post-blast survival period in exacerbating injury. It may thus be concluded that both multiple blasts along with longer survival periods contribute to neuronal injury.

These observations on swine are corroborated in human studies. A MRSI study on warfighters exposed to explosive blast in the battle field several months to years prior to imaging, and exhibiting symptoms of mTBI showed significant decreases in the ratios of NAA/Choline and NAA/Creatine in the hippocampus, providing evidence of neuronal loss in the hippocampus [6, 11]. The greater neuronal loss resulting from multiple exposures also has some support in human studies [6].

### Astrocytes activation

In the current study, astrocyte activation is seen in the group of single blast exposed animals at about 1 month (the earliest time point examined). In our earlier study on the Yorkshire pig model [5], astrocyte activation and proliferation was observed at 2 weeks post-blast also following a single blast-exposure. Thus, astrocyte activation is an early response to explosive blast. Compared to the single blast-exposed group, the doublet and triple blast-exposed animals with longer post survival times (6–8 months), had ~20–30% more activated astrocytes in the dentate hilus and molecular layer. Increased numbers of astrocytes were also clearly observed (though not quantified) also in CA1. The increases in astrocyte density in these areas may be in response to the neuronal injury also found in these areas of the hippocampus. Since no significant neuronal injury was observed in the hilus in the single blast-exposed group compared to controls, but an increased number of astrocytes were found, astrocyte activation may be an early trigger of the injury process in the hippocampus. In support of this possibility, proteomic analysis has confirmed that GFAP levels are dramatically elevated as early as 6 h post-blast in cerebrospinal fluid [3] and hippocampal tissue, suggesting an early activation of astrocytes.

Astrogliosis has been observed in small animal models of explosive blast [8, 22] as well as non-penetrating closed head injury models [17]. A recent histopathological study of brains obtained post-mortem from soldiers with a history of chronic and acute blast TBI also corroborate GFAP positive astroglial activation in the hippocampus [28] as an early response to blast. Despite the prominence of this cell type in traumatic brain injury, little is yet known as to its contribution to mild traumatic brain injury. A hypothesis yet to be tested, is that these activated astrocytes may play a role in inflammatory processes that lead to neuronal injury [3]. For instance, using proteomic studies of the hippocampus of swine exposed to blast Agosten and colleagues (unpublished data) have found, elevated expression levels of several inflammatory proteins. As Astrocytes are known to be able to release a number of proinflammatory and inflammatory molecules [7, 15], these findings lend support to the hypothesis that inflammatory processes may be triggered by blast.

### Microglial activation

Microglial activation in the blast exposed swine brain is not so widespread. Activated microglia were found mostly in major white matter areas such as the corpus callosum and central white matter areas. They were more readily seen in some animals with double and triple blast exposure at longer post mortem intervals (6–8 month). However, in animals in which activated microglia were observed there was no detectable axonal degeneration by way of immunostaining these same areas for β-APP [5]. In another histopathological study of post-mortem brains of soldiers with a prior history of blast exposure, patches of β-APP injured axons were associated with activated microglia (i.e., Iba-1 immunoractive) [26]. The role of activated microglia among white matter tracts in blast mTBI and mTBI in general remains unclear. The presence of activated microglia are commonly thought to reflect an ongoing inflammatory response, where microglia are releasing several pro- and anti-inflammatory cytokines, chemokines and other molecules that participate in inflammation [21, 30].

### Tau expression

Multiple concussions that professional athletes can experience are associated with a clinical condition described as chronic traumatic encephalopathy (CTE) [24]. More recently, CTE has also been suggested to be present in veterans exposed to explosive blast [9]. The pathological signs of CTE are thought to resemble those of Alzheimer’s Disease (AD) [19] and is classified as a neurodegenerative tauopathy. Tauopathy is a condition associated with hyperphosphorylated Tau proteins that aggregate to form neurofibrillary tangles (NFTs). Immunohistochemical localization of hyperphosphorylated Tau show that the protein tangles in CTE are similar to those in AD [27]. The report by Goldstein et al. [9] on the examination of four postmortem brains from subjects with a history of exposure to explosive blast describe the expression of phosphorylated Tau in these brains. Moreover, in a murine model exposed to blast in a blast tube there was expression of multiple phospho-Tau and cleaved Tau species in neurons as early as 24 h after blast, which persisted in the hippocampus for at least 30 days post-exposure [13].

Since phosphorylated Tau expression, has been implicated with explosive blast exposure, we investigated its expression along with amyloid-β by immunohistochemistry, in the present studies at short (~1 month) and long (6–8 month) post-blast intervals. There are several well characterized Tau antibodies [13], among which AT-8 (Ser202 & Thr181) and CP13 (Ser202) has been commonly used in human and animal studies [9, 13, 24]. This antibody, which we used in our study, is known to detect phosphorylated Tau in a variety of species ranging from fruit flies to humans and thus a reliable marker for Tau. We did not find evidence of phosphorylated Tau in our blast-exposed swine either at early or late post-blast times. Additionally, the two recent studies of post-mortem brains of soldiers [26, 28] also did not find phosphorylated Tau expression or amyloid-β plaques in them, even though one of these studies [26] used the entire panel of phosphorylated Tau antibodies used in the earlier study that reported evidence of phosphorylated Tau expression [9]. Though the study by Shively and co-workers [28] do report that one case in their chronic exposure group (Case 1) did express amyloid-β plaques and Tau pathology, the etiology of this case was different from their other cases. The subject was the oldest of the group with a complicated medical history – in addition to blast exposure the subject had an etiology of having played contact sports and had been in three motor vehicle accidents between the ages of 5 and 40 years, which occurred some 40 and 14 years respectively prior to death at age 45 years. In this case there may well be causes other than blast exposure for the observed Tau pathology, perhaps resulting from the long-term moderate to severe concussive injuries [16]. Thus compelling evidence is lacking for a role of tau pathology in blast mTBI.

## Conclusions

In summary, the studies reported in this paper provide clear evidence of small but statistically significant levels of neuronal loss in the brain, including areas such as the hippocampus that are important for cognitive function. This finding corresponds to similar findings in the blast-exposed human brain based on MRSI [6]. Additionally, we observed significant astrocyte activation comparable to that observed in other studies of both explosive blast and closed head traumatic brain injury [8, 17]. The role of such astrocyte activation remains an important area for investigation, particularly in regards to neuroinflammation. In our study, activated microglia were prominent in white matter tracts, and particularly in animals exposed to multiple blasts and at long post-blast intervals. Interestingly, this microglial activation was evident even though injured axons (i.e. β-APP positive) were not found in these areas. In general, microglial activation appears to be a delayed response but whether this activity may contribute to inflammation related injury mechanisms at even longer post-blast times, remains to be explored. Negative findings in this study were the absence petechial hemorrhages or other gross signs of vascular injury.
